RETRACTED

# Application of Multislice Spiral CT Imaging Technology in the Diagnosis of Patients with Chest Sarcoidosis

**DOI:** 10.1155/2021/2887639

**Published:** 2021-11-23

**Authors:** Hong-Fei Ma, Liang Chen

**Affiliations:** The First Hospital of Jilin University, Changchun, Jilin Province 130012, China

## Abstract

**Objective:**

To study the qualitative value of multislice spiral CT (MSCT) dynamic enhancement scanning for solitary nodules (SPN) of the chest.

**Methods:**

In this paper, 40 cases of chest nodules (including 25 cases of malignant nodules, 8 cases of inflammatory nodules, and 7 cases of benign nodules) were first scanned to determine the scope of nodules. At the two rates of 5 ml/s and 3 ml/s, CT dynamic enhancement scans were performed at the center of the nodule, and the CT values, peak enhancement (PH) and peak time (PT) before and after SPN enhancement, were recorded. It is mainly strengthened, with 80% (20/25) of net added value between 20 and 60 Hu, and 20% (5/25) >60 Hu or <20 Hu. The enhancement peak and peak time are (31.31 ± 10.62) Hu and 45 s, respectively. The time-density curve (T-DC) showed a slowly rising type; the inflammatory nodules were mainly severely strengthened, with a net increase of >40 Hu. The enhancement peak value is (49.25 ± 12.44) Hu, and the peak time is 80 s and 140 s. There is a characteristic of rising and falling and then rising in the curve.

**Conclusion:**

Multislice spiral CT dynamic enhancement scan reflects the dynamic characteristics of chest nodular blood flow, which can be used to noninvasively evaluate and diagnose SPN.

## 1. Introduction

Solitary nodules (SPN) in the lungs are round or irregular shaped lesions with a maximum diameter of no more than 3 cm and are not accompanied by atelectasis, satellite lesions, and local lymphadenopathy. The disease has been reported all over the world. The incidence is insidious and has a certain degree of self-healing, so the incidence rate statistics are relatively difficult, but at present, the incidence rate of females worldwide is slightly higher than that of males. In addition, the mortality rate of elderly patients is high and still growing, which deserves attention. Solitary nodules of the chest can be caused by different diseases, and the morphology of different diseases has superimposed performance, which makes a lot of confusion in clinical diagnosis. With the development of imaging technology, especially the improvement of CT resolution, the detection rate of SPN is getting higher and higher, but the identification of benign and malignant is always difficult. Due to the characteristics of high contrast and low X-ray absorption rate of lung tissue, low-dose CT scan of the chest can diagnose lung diseases. The detection, differential diagnosis, and follow-up of lung nodules are one of the important subjects of chest imaging diagnosis. At present, the domestic and foreign research on the application of low-dose CT in the chest mainly focuses on the sensitivity assessment of lung nodule detection, and it rarely involves study on the morphological characteristics of nodules.

RETRACTED

Examination technologies such as MSCT, with its thin layer and fast and powerful postprocessing functions, have further promoted its wide application in the clinic. The continuous development of equipment not only significantly improved the image quality of various postprocessing such as three-dimensional reconstruction but also expanded the scope of application. With the further improvement of the MSCT scanning method and the faster development of computer postprocessing functions, postprocessing technologies such as MSCT three-dimensional imaging have also been rapidly developed and continuously improved. For example, the simulated endoscope (CTVB) technology can obtain trachea and bronchus images that look exactly like those seen in real fiber bronchoscopes, which obviously expands the scope of image diagnosis. Traditional 3D reconstruction techniques include Surface Occlusion Display (SSD), Maximum Intensity Projection (MIP), Minimum Intensity Projection (MinIP), Multiplanar Reconstruction (MPR, CPR), and Volume Rendering (VR) technologies. The image quality has also been greatly improved, and the required reconstruction time has been shortened significantly. Comprehensive and effective use of the abovementioned various postprocessing imaging techniques and methods can accurately display the anatomical structure of the lesion and its adjacent tissue relationships, which can provide more diagnostic information. Based on the abovementioned research background, the author performed CT dynamic enhancement scanning on 40 cases of SPN, retrospectively analyzed its CT performance, and explored the clinical application value of dynamic enhancement in the differential diagnosis of SPN, benign and malignant [1].

## 2. Materials and Methods

### 2.1. Case Information

The data of 40 patients with chest nodules who were first diagnosed in our hospital from September 2004 to February 2007 were collected by multislice spiral CT (MSCT) dynamic enhancement scan data. None of the patients received antitumor treatment. There were 25 males and 15 females, aged 29–72 years, with an average age of 57 years. There was no cavity and calcification in the lesion. The diameter is 0.9–4.5 cm, 34 cases are ≤3 cm and 6 cases are >3 cm, and the average is 2.7 cm. The data were divided into three groups: malignant, inflammatory, and benign. There were 25 cases of the malignant group, including 9 cases of squamous cell carcinoma, 9 cases of adenocarcinoma (including 2 cases of bronchioloalveolar carcinoma), 1 case of large-cell carcinoma, small-cell carcinoma, and adenosquamous carcinoma, and 4 cases of unclassified lung cancer (puncture is low in 2 cases of differentiated carcinoma, and 2 cases of liver metastasis were found at the same time). All patients underwent surgical resection, CT-guided lung biopsy, and bronchoscopy within 1 week of CT examination; 8 cases were in the inflammatory group (including 1 case of bronchiectasis with infection confirmed by surgery), and the remaining 7 cases were clinically treated, and follow-up showed that the lesion disappeared or was significantly reduced; 7 cases were in the benign group, including 3 cases of tuberculoma, 2 cases of sclerosing hemangioma, 1 case of chondromas hamartoma and schwannomas. Among them, 6 cases were confirmed by surgery, and 1 case of tuberculoma was confirmed by shrinking CT examination after regular antituberculosis treatment.

RETRACTED

### 2.2. Equipment and Instruments

MSCT scanning and image postprocessing were performed using our HI speed 16-slice spiral CT machine. The scanning parameters were set as layer thickness 3–5 mm, reconstruction interval 1.5 mm, pitch 1–1.5 mm, tube voltage 120 kv, tube current 220 mAs, standard algorithm was used, and FOV 250–430 mm. Small nodular lesions were further scanned for local lesion targets. When the patient is breathing calmly in the supine position, we tried to complete the area of interest scan with one breath hold. After the scan, the axial image is reconstructed at 1.5–3 mm intervals, and the reconstructed image is transmitted to the ADW4.2 workstation for multilevel, respectively. Reconstruction (MPR) technology, minimum density projection (MinIP) technology, surface obscuration reconstruction (SSD) technology, volume rendering (VR) technology, CT virtual bronchoscopy (CTVB), and other postprocessing technologies were used. In short, according to different cases, selective complementary use of a variety of different postprocessing methods and detailed analysis of various malignant imaging features of lung cancer patients are carried out. The image reconstruction should be based on the axial image, and the original thin layer image is reconstructed with a layer thickness of 1.25 mm and a mediastinal window (window width of 350–450 Hu, window position of 40–50 Hu) [2].

### 2.3. Inspection Method

The patient was placed in a supine position, and a breath-holding scan was performed after deep inhalation; the scan ranges from the lung tip to the upper edge of the liver. When a mass is found, it can be selectively used to narrow the field of view, and thin-layer scanning is used to target scan the lesion. In the workstation, all patients suspected of central lung cancer were subjected to tracheal and bronchial multiplanar reconstruction and three-dimensional reconstruction. The latter included MinIP and SSD, etc., and 65 patients underwent bronchial virtual endoscopy; 43 patients underwent pulmonary artery CT vessels contrast (CTA), the contrast agent is a nonionic contrast agent, 80–120 ml each time, injected from the superficial vein of the left or right upper limb, and the injection rate is 3 ml/s; the scanning range is determined according to the lesion, and the volume data are transferred to the workstation. First, two-dimensional reconstruction including axial, sagittal, coronal, and multiplane reconstruction is used, and then MIP and SSD are used to reconstruct the pulmonary artery and vein system blood vessel images. The main points of various postprocessing imaging techniques of MSCT are as follows: First, according to the location and shape of the mass or nodule, the best reconstruction method is chosen, each limitation is complemented, and the reliability of diagnosis is improved. Two-dimensional reconstruction often uses MPR and CPR and pays attention to adjust the reconstruction layer thickness; one can start from the minimum value of 0 and then gradually adjust to a larger thickness and repeat multiple times, while paying attention to adjust the CT value (threshold), and finally choose the best effect image. Then, one can focus on the observation of the trachea and trachea protuberance, bilateral main bronchus, hilar mass, surrounding nodules in the lung, etc. Secondly, VR, MIP, and transparency (including tracheal and lung surface reconstruction) are used for three-dimensional reconstruction, mainly to observe the surface conditions of the large blood vessels, trachea, and bronchus in the lungs and the relationship between the lung mass and the pleura. Finally, CTVB was used to observe the conditions of the trachea, bronchus, and the surface morphology of some tumors.

RETRACTED

### 2.4. Spiral CT Imaging Principle

When the opening irradiated by the plane light wave is circular, the Fraunhofer diffraction image in the far field is a circular bright spot in the center, and the outer ring is surrounded by light and dark circular stripes. The intensity distribution of diffraction fringes on the receiving screen is

(1) $$\begin{array}{c} I_{P}=I_{0}{\left[\frac{2J_{1}\left(x\right)}{x}\right]}^{2}, \end{array}$$

where *J*_1_(*x*) is the first-order Bessel function and *x*=(2*aπ*  sin  *φ*/*λ*), where *λ* is the laser wavelength, *a* is the radius of the circular hole, and *φ* is the diffraction angle. When *J*_1_(*x*) = 0, the fringe minimum value can be obtained. In the center of the diffraction pattern is a bright spot (Airy spot), which concentrates about 84% of the light energy. Let the diameter of the central bright spot (i.e., the first dark ring) be *d*; as sin  *φ* ≈ *φ*=(*d*/2*f*′)=1.22(*λ*/2*a*),

(2) $$\begin{array}{c} d=1.22\frac{\lambda f^{\prime }}{a}. \end{array}$$

In the formula, *f*′ is the focal length of the converging lens. When *f*′ and *λ* are known, the radius *a* of the circular hole can be obtained from the abovementioned formula by measuring *d*. Therefore, measuring the size of the Airy disk or its changes can help precisely measure or analyze the size of the tiny inner hole [3].

The gap measurement method can calculate the gap width by measuring *xk* according to formula (2) and can also obtain the gap width by measuring the interval value between two dark stripes. When measuring displacement with the gap measurement method, that is, measuring the change amount *δ*=*b*′ − *b* of the slit width *b*, the absolute method can be used to find the two slit widths *b* and *b*′ before and after the change and then subtracted. One can also use the incremental method. The formula used in the latter is

(3) $$\begin{array}{c} \delta =b^{\prime }-b=\frac{k\lambda }{\sin\;\theta }-\frac{k^{\prime }\lambda }{\sin\;\theta }=\left(k-k^{\prime }\right)\frac{\lambda }{\sin\;\theta }=\Delta N\frac{\lambda }{\sin\;\theta }. \end{array}$$

In the formula, Δ*N*=*k*′ − *k* is to record the number of fringe changes through a fixed diffraction angle *θ*. Therefore, as long as Δ*N* is measured, the displacement value *δ* can be obtained. This situation is similar to the fringe count of an interferometer. The gap method as a sensitive optical sensor can be used to measure changes in various physical quantities, such as strain, pressure, temperature, flow rate, and acceleration.

Reflection diffraction is measured using the edge of the measured object and the slit formed by the mirror. The optical path difference where the dark streak *k* appears at the point is

(4) $$\begin{array}{c} 2b\;\sin\;\theta -2b\;\sin\left(\theta -\varphi \right)=k\lambda . \end{array}$$

In the formula, *θ* is the angle between the incident parallel laser beam and the reflector, and *φ* is the diffraction angle, which is the angle between the intersection of the slit and the mirror and the connection between point *P* and the reflected light that meets the law of reflection. Under the geometric relationship of the figure, the slit width can be expressed as

(5) $$\begin{array}{c} b=\frac{kL\lambda }{\left[2x_{k}\left(\cos\;\theta +\left(x_{k}/2L\right)\sin\;\theta \right)\right]}. \end{array}$$

Equation (5) shows that the measurement sensitivity has doubled due to reflection. Reflection diffraction technology is mainly used for surface quality assessment, linearity measurement, gap measurement, etc. This method easily realizes detection automation, and its detection sensitivity can reach 2.5–0.025 *μ*m.

RETRACTED

In actual measurement, it is often encountered that there is an interval *z* when the two sides forming the slit are not in the same plane. At this time, the diffraction pattern appears to be asymmetrical. The method of performing precise measurement using the diffraction fringes formed when the reference object and the measured object are not in the same plane is called the separation gap method. The measurement principle of the separation gap method is shown in Figure 1. By measuring the positions *x*_*k*1_ and *x*_*k*2_ of the dark stripes on positive and negative orders *k*_1_ and *k*_2_, the slit width *b* and interval *z* can be calculated by the following formula:

(6) $$\begin{array}{c} b=\frac{k_{1}L\lambda }{x_{k1}}-\frac{zx_{k1}}{2L}=\frac{k_{2}L\lambda }{x_{k2}}+\frac{zx_{k2}}{2L}. \end{array}$$

### 2.5. Statistical Methods

On the mediastinal window of the flat scan and dynamic enhanced scan sequence images, the CT values of the center of the lesion and the thoracic aorta (the upper part of the aortic arch is replaced by the brachial artery) are measured. The region of interest (ROI) is chosen as large as possible to reduce noise, and attention is paid to avoid liquefaction and necrosis to reduce part of the volume effect. The CT net added value (post-enhancement-level scan) of each period is calculated, and the enhancement peak (PH) and peak time (PT) are recorded. The m-group and inflammatory group were statistically analyzed by the *t*-test, with *P* < 0.05 being statistically significant. The benign group was not statistically processed due to the complex disease type (the dynamic enhancement mode was quite different).

## 3. Results

### 3.1. CT Net Value-Added, PH, and PT before and after SPN Enhancement

The net increase value of the malignant group was 12.8–70.0 Hu, PH value: (31.31 ± 10.62) Hu, and PT value: 45 s; the net increase value of the inflammatory group was 41.1–72.9 Hu, PH value: (49.25 ± 12.44) Hu, and PT value: 80 and 140 s, appearing twice. There was a significant difference between the malignant group and the inflammatory group after augmentation in 45, 60, 80, 120, and 140 s (*P* < 0.05, and *t* values were 3.0273, 4.0339, 3.8210, 2.5568, and 2.8992). The net increase in the benign group was 15.7 to 59.7 Hu (Table 1) [4].

RETRACTED

### 3.2. The Effect of Contrast Agent Enhancement at Different Rates on SPN and Large Blood Vessels and Its T-DC

Bolus injection rates of 5 and 3 ml/s, respectively, were used. In 25 cases of malignant nodules, using 5 ml/s (7 cases) and 3 ml/s (the remaining 18 cases), the net value-added value of each period observed was not statistically significant (*P* value >0.05), and T-DC data were combined into 25 cases. The contrast value enhancement of the contrast agent at different rates showed a net increase in the main A (or head and arm A) at various times. After enhancement, 15, 45, 60, 120, 140, and 160 s were statistically significant (*P* < 0.05, and *t* values were 2.2946, 2.1534, 3.6037, 2.2428, 3.0469, and 3.2124), and there is no statistical difference between the two when the peak value of 30 s is enhanced. The malignant group first rose to a peak at a moderate rate and then rose slightly after maintaining a certain level during the study period; the inflammatory group first rose quickly and then rose slightly, then slowly rose near the peak level, and after a certain degree, fell to moderate. The speed rises to the peak and then falls close to the original inflection point. The level rises slowly, forming two similar peaks within the study range (Figure 2). The T-DC in the inflammatory and malignant group is similar to that reported by Zhang Miming and others. In the benign group, the curve of sclerosing hemangioma is similar to that of malignant nodules, but the increase is larger; the curves of tuberculoma and schwannomas are low and flat, and the T-DC of hamartoma is slightly higher than that of schwannomas. The aorta (or brachial artery) enhanced at different rates has a similar T-DC morphology, and all form steep peaks within 30 seconds. The high-rate curve is always at the top of the graph (Figure 3) [5].

### 3.3. SPN Enhancement Mode

The enhancement pattern of SPN is more complicated. In the malignant group, 8% (2/25) showed uniform enhancement; 92% (23/25) showed uneven enhancement or even enhancement over time, of which 2 cases simultaneously showed surrounding enhancement (Figure 4); 6/8 in the inflammatory group showed peripheral enhancement (including circular enhancement around the liquefied necrotic focus); 2/8 showed uniform enhancement (Figure 5); 4/7 cases in the benign group showed uneven strengthening (Figure 6), and 3/7 showed the strengthening of the envelope [6].

## 4. Discussion

### 4.1. Certain Differences in the Net Value-Added of SPNs with Different Properties in the Dynamic Enhanced Scan

The inflammation and malignant nodules had a statistically significant difference in net value increase after 45 to 80 s and 120 to 140 s after enhancement. After the intravenous injection of the contrast agent, it first relies on the blood vessel to transport to the tissue. The early contrast agent enhancement is mainly formed by the contrast agent in the blood vessel. As time goes on, the contrast agent gradually diffuses from the blood vessel to the outside of the blood vessel to the later tissue. Contrast enhancement is accomplished by intravascular and extravascular contrast agents. The different histology of SPN and the different characteristics of microvessel formation in nodules make this hemodynamic model have some differences, and the SPN enhancement CT net value-added has certain differences. The work in [4] reported that the net value-added of malignant nodules is lower than that of inflammatory nodules and higher than that of benign nodules. The diagnostic index of malignant nodules is 20–60 Hu; domestic scholars report that the net value-added of malignant nodules is mostly 20–60 Hu. In the past, a few were >60 Hu or <20 Hu, most of the pneumonia nodules were >60 Hu, and a few were between 20 and 60 Hu. This group of 40 case studies shows that malignant nodules are close to that mentioned above, and inflammatory nodules are all >40 Hu, which may be related to the multicellular composition of inflammation and at different pathological stages. MSCT and image postprocessing technology images show that the basic malignant signs of peripheral lung cancer mainly include lobulated sign, burr or spinous protrusion on the edge, vacuole sign, pleural depression sign, vascular bundle sign, bronchial inflation sign, cancerous cavity sign, and significantly enlarged lymph nodes (diameter >1.0 cm) in the mediastinum spread to distant tissues and organs.

RETRACTED

There are differences in PT between the malignant group and inflammatory group. The work in [5] shows that the contrast agent flow rate is 4.0 ml/s, and the average peak enhancement time of chest malignant lesions is 60 s. At the same time, it shows that the enhancement peak of most lung cancer is within 1 min (4 ml/s, 100 ml). The study in [6] shows that the PT of malignant nodules is earlier than that of inflammatory nodules. The data in this group showed that malignant nodules' PT appeared in 45 s and inflammatory nodules' PT appeared later and appeared twice in 80 s and 140 s. The inflammatory group had higher nodular enhancement in the 45–80 s and 120–140 s two-stage relative malignant groups. From 45 to 80 s, the contrast agent diffused from inside to outside. From 120 to 140 s, contrast enhancement is maintained by intravascular and extravascular contrast agents. The thicker and straight capillaries of inflammatory nodules have more blood perfusion in the early stage of enhancement than the immature tumor capillaries of malignant nodules, and the result of secondary vascular circulation in the nodules may appear in the later stage [7].

### 4.2. Significance of T-DC

SPN's T-DC reflects the kinetic changes of the contrast agent in the nodules. Different forms of T-DC in good and bad nodules indirectly showed the difference in tissue blood supply, extracellular fluid volume, and contrast agent diffusion characteristics. There are a large number of interstitial spaces in malignant nodules, the permeability of immature tumor capillaries is increased, and the lymphatic vessels are significantly reduced or absent. Therefore, the malignant group has a moderate increase in T-DC. The outflow is generally slower than in normal tissues, and there is still a delay in the late rise. However, there are dilated capillaries in the inflammatory nodules, the diameter of the tube is generally more uniform, the direction is regular, the drainage lymph is more normal, and the T-DC rises near the peak and then drops to a certain level and then rises. Also, the combined effect of factors such as the second cycle is seen [8].

The T-DC of large vessels showed that the contrast curves of the large vessels showed similar enhancement curves, and the high flow rate T-DC was always located above. With high flow rate per unit time perfusion of large vessels, large vessels always have a high CT net added value, the contrast of blood vessels and surrounding tissues and lesions is increased, and the resolution of CT images is higher. After enhancement, 45–60 s and 120–160 s can improve the image quality.

### 4.3. SPN Enhancement Mode

The strengthening mode of SPN refers to its strengthening structure and method. The difference of strengthening mode directly reflects the difference of blood vessel density inside the nodules. The work in [8] shows that malignant nodules are uniformly strengthened or from uneven to evenly strengthened, accounting for 79.3%. Inflammatory nodules are mostly strengthened around. Most of the malignant nodules in this group are unevenly enhanced (including surrounding enhancement and uniform enhancement over time), and a few are always uniformly enhanced. The image performance is related to the size of the nodules. The bigger the nodules are, the higher the performance. Inflammatory nodules have different durations, various tissue components, and a greater degree of enhancement, mainly surrounding enhancement, and a few are uniformly enhanced. In benign nodules, tuberculous tuberculosis is composed of fibrous encapsulated cheese necrotic tissue, which is mainly manifested by enhanced capsule. The sclerosing hemangioma is unevenly strengthened, and the pathological basis may be caused by the cavernous hemangioma-like tissue in the lesion. Schwannomas and hamartomas show mildly uneven enhancement.

RETRACTED

## 5. Conclusions

In summary, the application of CT in patients with atypical chest sarcoidosis can be used to more clearly observe the lesions, which is beneficial to the location, differentiation, and diagnosis of sarcoidosis lesions and has great clinical value.

## Figures and Tables

**Figure 1:** Schematic diagram of the separation gap method.

**Figure 2:** T-DC curve of malignant nodules and inflammatory nodules.

**Figure 3:** T-DC curves of the aorta at different rates.

**Figure 4:** Plain scan and dynamic enhanced scan image of the left lower lobe nodule.

**Figure 5:** Plain and dynamic enhanced scan images of inflammatory nodules in the right lower lobe.

**Figure 6:** Left lung lobe nodule plain scan and dynamic enhanced scan image.

**Table 1:** Changes in CT values before and after enhancement of malignant and inflammatory nodules.

	Flat sweep	15 s	30 s	45 s	60 s	80 s	100 s	120 s	140 s	160 s
Malignant nodules	38.52 ± 4.95	42.62 ± 9.43	63.62 ± 17.36	69.83 ± 16.28	65.44 ± 13.33	66.21 ± 13.38	64.40 ± 15.00	65.52 ± 16.79	67.42 ± 16.35	63.95 ± 14.23
Inflammatory nodules	42.93 ± 9.18	53.48 ± 15.77	76.54 ± 12.62	87.85 ± 11.75	88.76 ± 10.81	90.75 ± 11.33	81.74 ± 15.94	85.09 ± 9.06	91.18 ± 15.70	79.94 ± 16.71

## Data Availability

The data used to support the findings of this study are available from the corresponding author upon request.
